# Responses of apoptosis and matrix metabolism of annulus fibrosus cells to different magnitudes of mechanical tension *in vitro*

This article has been retracted.

**DOI:** 10.1042/BSR20182375

**Published:** 2019-02-22

**Authors:** Yanhai Jiang, Lianqiang Fu, Yeliang Song

**Affiliations:** Department of Orthopaedics, The Affiliated Weihai Second Hospital of Qingdao University, Weihai 264200, China

**Keywords:** annulus fibrosus, cell apoptosis, intervertebral disc degeneration, matrix, mechanical tension

## Abstract

Background: Annulus fibrosus (AF) is important to confine disc nucleus pulposus (NP) tissue during mechanical load experience. However, the knowledge on AF cell biology under mechanical load is much limited compared with disc NP. Objective: The present study aimed to investigate responses of apoptosis and matrix metabolism of AF cells to different magnitudes of mechanical tension *in vitro*. Methods: Rat AF cells were subjected to different magnitudes (5, 10, and 20% elongations at a frequency of 1.0 Hz for 6 h per day) of mechanical tension for 7 days. Control AF cells were cultured without mechanical tension. Cell apoptosis ratio, caspase-3 activity, gene/protein expression of apoptosis-related molecules (Bcl-2, Bax, caspase-3/cleaved caspase-3 and cleaved PARP), matrix macromolecules (aggrecan and collagen I) and matrix metabolism-related enzymes (TIMP-1, TIMP-3, MMP-3, and ADAMTS-4) were analyzed. Results: Compared with 5% tension group and control group, 10 and 20% tension groups significantly increased apoptosis ratio, caspase-3 activity, up-regulated gene/protein expression of Bax, caspase-3/cleaved caspase-3, cleaved PARP, MMP-3, and ADAMTS-4, whereas down-regulated gene/protein expression of Bcl-2, aggrecan, collagen I, TIMP-1, and TIMP-3. No significant difference was found in these parameters apart from Bcl-2 expression between the control group and 5% tension group. Conclusion: High mechanical tension promotes AF cell apoptosis and suppresses AF matrix synthesis compared with low mechanical tension. The present study indirectly indicates how mechanical overload induces disc degeneration through affecting AF biology.

## Introduction

Intervertebral disc is a cartilaginous structural which degenerates much earlier than other tissues in life [1]. Disc degeneration often results in unfortunate consequences, such as low back pain, sciatica, and other distressing and costly spinal disorders [2]. Though lots of findings on its pathogenesis of disc degeneration have been found, there are still some important points remaining unclear.

The etiology of disc degeneration is multifactorial. Though genetic factors [3] and ageing [1] are known as predisposing factors of disc degeneration, mechanical loading plays a role in regulating disc biology during disc degeneration [4–14]. The intervertebral disc contains three parts: the central nucleus pulposus (NP), the peripheral annulus fibrosus (AF), and cartilage endplates (CEP) [15]. During daily activities, the disc NP region plays an important role in absorbing and transmitting mechanical load [16]. However, disc AF tissue also is a key element for maintaining disc function. It confines the compressed NP tissue during mechanical loading experience [17]. In the degenerated disc tissue, some structural changes including tears and fissures are common [18,19]. However, the knowledge on AF cell biology under mechanical load is limited until now.

Because disc structure is closely related with cellular bioactivity and matrix metabolism, further understanding on cellular and compositional alterations may be important to understand disc mechanobiology in health and disease [20]. Importantly, increased cellular apoptosis and imbalance of matrix metabolism are two classical features of the degenerative disc tissues [21,22]. Therefore, in the present study, we mainly aimed to investigate cell apoptosis and matrix metabolism of AF cells under different magnitudes of mechanical tension.

## Materials and methods

### Ethical statement

Thirty-seven healthy Sprague–Dawley rats (10–11 weeks old, 360–380 g weight) were used in the present study. All animal procedures were strictly performed according to relevant guidelines of Ethical Committee of Qingdao University [SHNK(E) 2011-021].

### AF cell isolation and culture

Briefly, the spinal column was separated after the rats were killed by excessive carbon dioxide inhalation. Then, AF tissue samples were collected and washed with sterile phosphate-buffer solution (PBS). To obtain cell pellets, AF tissue was respectively digested by 0.25% trypsin (Gibco, U.S.A.) for 3–5 min and 0.2% type I collagenase (Gibco, U.S.A.) for 15–20 min at 37°C. Subsequently, AF cell pellets were re-suspended in Dulbecco’s modified Eagle’s medium (DMEM) supplemented with 10% FBS (Gibco, U.S.A.) in a 5% CO_2_ incubator. When approximately 80% confluence was reached, AF cells were dismissed using 0.25% trypsin solution and then subcultured. The passage 3–4 AF cells were used in each assay in the present study. To investigate responses of AF cells to different magnitudes of mechanical tension, AF cells were seeded on to the flexible silicone membrane affiliated to the culture chamber of an FX-5000T Flexercell tension plus system (Flexcell International Corp.) and subjected to different mechanical tensions (5, 10, and 20% elongation) at a frequency of 1.0 Hz for 6 h per day for 7 days. The magnitudes of mechanical tension were designed according to our own criteria and a previous study [23].

The control AF cells were kept in static culture. Culture medium was replaced by fresh medium every 3 days.

### Flow cytometry

After 7 days of culture, both adherent and suspended NP cells were collected and washed with PBS for three times to remove redundant FBS in the culture medium. Then, 1 × 10^5^ cells in each group were sequentially re-suspended in 195 μl Annexin V-PE binding buffer and stained by 5 μl Annexin V-PE solution for 20 min under dark conditions. Then, the prepared AF cells were subjected to a flow cytometer (Beckman-Coulter, Pasadena, CA, U.S.A.), and cell apoptosis ratio was analyzed by a FlowJo software (FlowJo LLC, Ashland, OR, U.S.A.).

### Caspase-3 activity

After 6 days of culture, both adherent and suspended NP cells were collected as described above. Then, caspase-3 activity was measured using a Caspase-3 Activity Detection Kit (Beyotime, China). Briefly, AF cells were lysed using the lysis buffer in the kit. Then, a reaction system containing the supernatant was used to read the optical density (OD) value at a wavelength of 405 nm. Finally, caspase-3 activity (U) was calculated according to a standard curve created using *p*NA in the kit.

### Real-time PCR

Briefly, AF cells were collected as described above. The total RNA samples were extracted using the TRizol reagent (Invitrogen, U.S.A.) and reverse-transcribed into cDNA templates using a SuperRT cDNA Synthesis Kit (CWBio, China) according to the manufacturer’s instructions. Then, real-time PCR was performed on a reaction system consisting of cDNA templates, primers (Table 1) and SYBR Green Mix (CWBio, China). PCR amplications were performed according to the protocol: 95°C for 5 min, followed by 40 cycles of 95°C for 10 s, 55°C for 10 s, and 72°C for 20 ss. *GAPDH* was used as a reference gene. Relative gene expression of target molecules was calculated with the method of 2^–ΔΔ*C*^_t_.

**Table 1:** Primers of target genes

Gene	Forward (5′–3′)	Reverse (5′–3′)
*GAPDH*	CCATCAACGACCCCTTCATT	ATTCTCAGCCTTGACTGTGC
*Aggrecan*	GCCTGCAAGGGAAATGTGTG	GGCGGAAAGATTTGCCGTTAG
*Collagen II*	GACCTCCGGCTCCTGCTCCTCTTAG	GACAGCACTCGCCCTCCCGTTTTTG
*Bax*	GGCGAATTGGCGATGAACTG	CCCAGTTGAAGTTGCCGTCT
*Bcl-2*	CGCCCGCTGTGCACCGAGA	CACAATCCTCCCCCAGTTCACC
*Caspase-3*	TACCCTGAAATGGGCTTGTGT	GTTAACACGAGTGAGGATGTG
*TIMP-1*	ACCTGGTTAAGGGCTAAATTCATG	ATTTCCACAGCGTCGAATC
*TIMP-3*	CCTTTGGCACTCTGGTCTACACT	CTTTCAGAGGCTTCCGTGTGA
*MMP-3*	AAAGAACCCGCTGAGAGCAG	AACCTCCATGCCAGCATCTT
*ADAMTS-4*	CGTTCCGCTCCTGTAACACT	TTGAAGAGGTCGGTTCGGTG

### Western blot

AF cells were collected as described. Total protein was extracted using RIPA Lysis Buffer (CWBio, China). Protein concentration was determined using a BCA Protein Assay Kit (CWBio, China). Then, equal protein samples in each group were separated by SDS/PAGE and transferred on to the nitrocellulose membranes. The nitrocellulose membranes were blocked by 5% BSA and then incubated with primary antibodies (GAPDH: CW0100, CWBio, China; aggrecan: NB120-11570, Novus, U.S.A.; Collagen I: ab90395, Abcam, U.S.A.; Cleaved caspase-3: #9664, Cell Signaling Technology, U.S.A.; Cleaved PARP: #5625, Cell Signaling Technology, U.S.A., all diluted at 1:1000). After washing with TBS containing 0.1% Triton X-100 (TBST) for 15 min, the nitrocellulose membranes were incubated with corresponding secondary antibodies for 1 h at room temperature. Finally, protein bands on the membranes were visualized using an eECL Western Blot Kit (CWBio, China) and analyzed using ImageJ software.

### Statistical analysis

All data were expressed as mean ± S.E.M. Each experiment was performed for three times. For comparisons between groups, the one-way ANOVA and least significant difference (LSD) assay were performed using SPSS 19.0 software (International Business Machines Corp., Amonk, NY, U.S.A.).

## Results

### Cell apoptosis ratio

Though cell apoptosis ratio between the control group and 5% tension group showed no significant difference, 10% tension group and 20% tension group showed a significant increase in cell apoptosis ratio compared with the control and 5% tension group in a tension magnitude-dependent manner, with a higher apoptosis ratio in the 20% tension group than in the 10% tension group (Figure 1).

**Figure 1:** Cell apoptosis analysis AF cell apoptosis ratio under different magnitudes (5, 10, and 20% elongations) of mechanical tension was analyzed by flow cytometry. Data are presented as mean ± S.D. (*n*=3). *: Indicates a statistical difference (*P*<0.05) between two groups.

### Caspase-3 activity

Our results showed that caspase-3 activity in the control group is similar to that in the 5% tension group. However, 10% tension group and 20% tension group showed a significant increased caspase-3 activity compared with the control and 5% tension groups in a tension magnitude-dependent manner, with a higher caspase-3 activity in the 20% tension group than in the 10% tension group (Figure 2).

**Figure 2:** Caspase-3 activity analysis Caspase-3 activity of AF cells under different magnitudes (5, 10, and 20% elongations) of mechanical tension was analyzed. Data are presented as mean ± S.D. (*n*=3). *: Indicates a statistical difference (*P*<0.05) between two groups.

### Expression of apoptosis-related molecules

Here, we analyzed gene expression of Bcl-2, Bax, and caspase-3, and protein expression of cleaved caspase-3 and cleaved PARP to evaluate cell apoptosis. Results showed that no significant difference was found in the expression of these molecules between the control group and 5% tension group apart from the significantly up-regulated gene expression of Bcl-2 in the 5% tension group. However, 10% tension group and 20% tension group significantly increased gene/protein expression of Bax, caspase-3, cleaved caspase-3, and cleaved PARP whereas decreased gene expression of Bcl-2 compared with the control group and 5% tension group. Moreover, a tension magnitude-dependent manner was found between the 10% tension group and 20% tension group (Figure 3).

**Figure 3:** Expression of apoptosis-related molecules Gene/protein expression of Bcl-2, Bax, caspase-3/cleaved caspase-3, and cleaved PARP in AF cells under different magnitudes (5, 10, and 20% elongations) of mechanical tension was analyzed. (**A**) Real-time PCR analysis. (**B**) Western blot analysis. Data are presented as mean ± S.D. (*n*=3). *: Indicates a statistical difference (*P*<0.05) between two groups.

### Expression of matrix molecules

Both gene expression and protein expression of matrix macromolecules (aggrecan and collagen I) were analyzed to evaluate matrix biosynthesis of AF cells. Results showed that both gene expression and protein expression of them in the 10% tension group and 20% tension group were significantly decreased compared with the control and 5% tension group in a tension magnitude-dependent manner. However, 5% tension group showed similar expression of these molecules compared with the control group (Figure 4).

**Figure 4:** Expression of matrix macromolecules Gene and protein expression of aggrecan and collagen I in AF cells under different magnitudes (5, 10, and 20% elongations) of mechanical tension was analyzed. (**A**) Real-time PCR analysis. (**B**) Western blot analysis. Data are presented as mean ± S.D. (*n*=3). *: Indicates a statistical difference (*P*<0.05) between two groups.

### Expression of matrix metabolism-related enzymes

Gene expression of TIMP-1, TIMP-3, MMP-3, and ADAMTS-4 was analyzed to evaluate matrix anabolism and matrix catabolism. Results showed that gene expression of MMP-3 and ADAMTS-4 significantly or non-significantly increased compared with those in the control group in a tension magnitude-dependent manner. No significant difference in the expression of TIMP-1 and TIMP-3 was found between the control group and 5% tension group, whereas their expressions in the 10% tension group and 20% tension group were significantly decreased compared with the control group and 5% tension group (Figure 5).

**Figure 5:** Expression of matrix metabolism-related enzymes Gene expression of TIMP-1, TIMP-3, MMP-3, and ADAMTS-4 in AF cells under different magnitudes (5, 10, and 20% elongations) of mechanical tension was analyzed by real-time PCR. Data are presented as mean ± S.D. (*n*=3). *: Indicates a statistical difference (*P*<0.05) between two groups.

## Discussion

Disc degeneration encompasses a series of anatomic changes that contribute to musculoskeletal disorders. The intervertebral disc allows for load support and spinal flexibility and is exposed to substantial mechanical demands during daily activities. However, these mechanical demands are reported to be initiating factors for disc degeneration in some cases [16]. Recently, increasing evidence has indicated that cell-mediated matrix remodeling is the secondary response to mechanical stimulation during daily activities, which ultimately leads to degenerative changes [8,12,13,24–26]. For intervertebral disc, much progress has been made in explaining mechanobiologic effects of NP tissue, whereas much less has been done in investigating biological responses of AF tissue to mechanical stimuli. Further understanding on AF mechanobiology is also of great significance to elucidate mechanical load-related disc degeneration.

Under physiological conditions, AF tissue experiences transverse tension resulted from NP swelling [17]. The present study mainly investigated responses of apoptosis and matrix metabolism of AF cells to mechanical tension *in vitro*. Our results showed that high mechanical tension promoted AF cell apoptosis and suppressed AF matrix homeostasis compared with the low mechanical tension. In light of that increased cell apoptosis and imbalanced matrix metabolism are two features of degenerative disc tissue [27], this study helps us understand AF biology better under mechanical tension and provides some basic knowledge about mechanical load-related disc degeneration.

Adequate disc cell number within the disc tissue is important to refresh and synthesize matrix proteins [21,28,29]. Decrease in cell number due to cell death aggravates and accelerates disc degeneration. Though several studies have investigated disc NP cell apoptosis under mechanical stimulation [6–10,13,25], no study has investigated AF cell apoptosis under mechanical tension. Here, we found that high mechanical tension significantly increased cell apoptosis ratio and caspase-3 activity, up-regulated gene/protein expression of Bax, caspase-3, cleaved caspase-3, and cleaved PARP, and down-regulated gene expression of Bcl-2 in AF cells compared with the low mechanical tension and control group, indicating that high mechanical tension promotes AF cell apoptosis compared with the low mechanical tension. This is in-line with previous opinion that high mechanical load promotes disc degeneration [16].

AF tissue structural changes including tears and fissures are common in the degenerated disc [18,19]. Matrix homeostasis is important for the maintenance of structural integrity [16,30], however, the knowledge on AF cell biology under mechanical load is limited until now. In the present study, we found that high mechanical tension significantly decreased expression of matrix molecules (aggrecan and collagen I) in AF cells compared with the low mechanical tension, indicating that high mechanical tension inhibits matrix production compared with the low mechanical tension. Furthermore, high mechanical tension significantly up-regulated gene expression of MMP-3 and ADAMTS-4, whereas down-regulated gene expression of TIMP-1 and TIMP-3 in AF cells compared with the low mechanical tension, indirectly suggesting again that high mechanical tension facilitates matrix catabolism and suppresses matrix anabolism.

In the present study, we also found that some parameters evaluating cell apoptosis and matrix metabolism between the control group and 5% tension showed no significant difference. This indicates that there may be an appropriate magnitude of mechanical tension that can maintain/improve normal bioactivities of AF cells. Previously, several studies have also demonstrated a threshold of mechanical compression for disc biology [4,31]. To further investigate the mechanical tension’s ‘window effect’, more investigations are needed. The present study also has several limitations. First, there are some other changes (i.e. cell senescence and inflammation response) during disc degeneration [32,33], we just focussed on cellular apoptosis and disc matrix metabolism in the present study, Second, the present study is just an observational research. We will further investigate signaling transduction pathways behind this process in the future research plan. Third, though AF region mainly experiences mechanical tension, it is also subjected to some mechanical compression to some extent. However, the present study only observed AF biological changes under mechanical tension.

## Conclusion

Together, the present study investigated the responses of apoptosis and matrix metabolism of AF cells to different mechanical tensions. Our results showed that high mechanical tension promotes AF cell apoptosis and suppresses AF matrix synthesis compared with the low mechanical tension. The present study first sheds a light on AF cell apoptosis and matrix metabolism under mechanical tension, and indirectly indicates that high mechanical tension can induce disc degeneration through affecting AF biology.

## Abbreviations

AF: annulus fibrosus
GAPDH: glyceraldehyde-3-phosphate dehydrogenase
MMP: matrix metalloproteinase
NP: nucleus pulposus
PBS: phosphate-buffer solution
TIMP: tissue inhibitor of metalloproteinase 1
